The article "Exploring the link between economic policy uncertainty, financial development, ecological innovation and environmental degradation; evidence from OECD countries" was retracted in 2025. Reasons: unreliable results or conclusions; concerns about the article.

# Exploring the link between economic policy uncertainty, financial development, ecological innovation and environmental degradation; evidence from OECD countries

**DOI:** 10.1371/journal.pone.0307014

**Published:** 2024-09-11

**Authors:** Xiaowei Zheng, Muhammad Faheem, Khusniddin Fakhriddinovch Uktamov

**Affiliations:** 1 Business School, Suzhou University, Suzhou, China; 2 Schools of Economics, Bahauddin Zakaryia University, Multan, Pakistan; 3 International School of Finance and Technology, Tashkent, Uzbekistan; Universiti Malaysia Sabah, MALAYSIA

## Abstract

Governments have been concerned with balancing economic growth and environmental sustainability. Nevertheless, it has been noted that sustainable development is interconnected with economic variables, the institutional framework, and the efficacy of ecological regulatory measures. This study experimentally examines the correlation of economic policy uncertainty (EPU), financial development (FD), ecological innovation (EI), corruption (IQ), foreign direct investment (FDI), trade openness (TR), natural resource rent (NRR), and CO_2_ emission. We utilized longitudinal data from the Organization for Economic Cooperation and Development (OECD) countries from 2003 to 2021 to address the existing research void. This study used sequential processes of the linear panel data model (SELPDM) and the SYS-GMM approaches in obtaining consistent and efficient results. The inverse U-shaped relationship between FD and environmental degradation (ED) is confirmed by the long-term elasticity estimates generated by the SELPDM method Elasticity estimates for the long-run show that rigorous ecological regulations, higher renewable energy utilization, higher FD and less corruption, an interaction between FD and rigorous ecological regulations all contribute to reduced ED. Its also being observed that both EPU, FDI and trade openness are positively affecting the ED. It confirms the idea of pollution refuge between the OECD countries. The causality test results show that corruption and FD had reciprocal links with ED, while FDI, trade openness and strict environmental policies were also found to have bidirectional linkage with ED. To achieve sustainable development and prevent environmental degradation in the long term, we propose implementing an institutional financial framework and FD in OECD nations. This may be accomplished by focusing on the effectiveness of environmental regulatory laws and creating a conducive institutional environment.

## 1. Introduction

Degradation of the natural environment is now widely recognized as a significant threat to the long-term prosperity of nations of all economic levels. Carbon dioxide (CO_2_) and other greenhouse gases contribute to the depletion of the ozone layer and are the primary drivers of environmental degradation (ED). One of the SDGs’ goals is to reduce greenhouse gas emissions [1]. Climate change and worldwide degradation of ecological quality directly result from human-caused CO_2_ emissions, producing global warming. Therefore, it is essential to learn what aspects contribute to CO_2_ emissions. Because it encourages manufacturers to stick with inefficient and potentially dangerous production practices, economic policy uncertainty (EPU) can raise CO_2_ emissions [2]. High EPU may also cause a rise in CO_2_ emissions by discouraging R&D, innovations, and the usage of renewable energy (RE) sources. In addition, businesses in the high EPU era may exploit the natural environment for private gain because of lax enforcement of norms and regulations [3]. Zhou et al. [4] believe that political stability could serve as a stimulus for addressing the environmental degradation problem caused by EPU. Reducing waste, stopping pollution, and protecting the environment are all aims of stable governments. Maintaining peace in government and a consistent set of policies can reduce pollution. Therefore, to provide solutions to environmental deterioration, it is necessary to study the correlation between EPU and CO_2_ emissions in the context of ecological degradation.

The article "Exploring the link between economic policy uncertainty, financial development, ecological innovation and environmental degradation; evidence from OECD countries" was retracted in 2025. Reasons: unreliable results or conclusions; concerns about the article.

Economic policy uncertainty also affects climate change matters by means of regulatory mechanisms that promote openness in the financial sector to reduce the impact of climate change [5]. The EPU’s use of inadequate valuation techniques for investments and output potential of climate change projects may jeopardize the achievement of climate targets, leading to disruptions in climate policy operational programs. Academic experts affirm the importance of EPU (Fossil Fuel Phase-Out) and the potential obstacles associated with climate change mitigation efforts [6]. According to Zhao et al. [7], EPU reduction regulations can affect investors that are looking to invest in green energy, causing a spillover impact.

When the EPU index rises, businesses and consumers delay or cut back on spending, hire new employees, and expand their operations. It was also found that taxes, spending, and monetary and regulatory policies were the media’s most common sources of policy uncertainty. This investigation aims to provide a picture of the interplay between policy ambiguity, the energy emission nexus, and the environmental Kuznets curve hypothesis. Du et al. [8] argued that EPU unquestionably influences the outside business environment, which impacts economic agents’ policy-making process. However, earlier studies overlooked the link between carbon emissions and EPU. This has a domino effect on carbon emissions because it influences microeconomic agents’ choices about their production [9]. According to OECD standards, the United States’ EPU index is relatively constant and stable. At times when the US EPU index is highest, for instance, total carbon emissions are also at their highest; conversely, when the EPU index is lowest, total carbon emissions are at their lowest. The result is that the government’s focus has shifted from environmental governance to the essential causes of the rise in the financial policy uncertainty index [10]. If the United States were to withdraw from the Paris Agreement, the EPU index would rise, and efforts to reduce carbon emissions would be given lower priority as a result [11]. This parallel suggests that the EPU will impact the environmental Kuznets curve hypothesis since the EPU will have a meaningful influence on the production and consumption of renewable and non-renewable energy sources. As a result, people spend less and save more steadily during times of low uncertainty and more and more during times of high uncertainty. A low EPU is thus associated with a rapid approach to the apex of the EKC, while a high EPU is associated with locations further from the apex.

The article "Exploring the link between economic policy uncertainty, financial development, ecological innovation and environmental degradation; evidence from OECD countries" was retracted in 2025. Reasons: unreliable results or conclusions; concerns about the article.

Recent studies indicate that the progress of financial systems has a range of effects on the environment. There are primarily two significant perspectives on the impact of financial growth on environmental sustainability [12]. A sophisticated financial system facilitates convenient access to capital, hence promoting investment. Consequently, the economy prospers, but simultaneously, energy consumption exacerbates environmental degradation. A well-functioning financial sector has the potential to offer financial support for cutting-edge technology and facilitate the implementation of energy-efficient manufacturing techniques [13], thereby mitigating environmental degradation. Additionally, financial markets can allocate funds for renewable energy projects and research and development expenses. Moreover, they can attract multinational corporations that can introduce sustainable technology to the country in which they operate [14]. Having a strong financial sector is essential for promoting economic advancement. However, it is also important to consider the environmental consequences that come with financial development. Over the course of historical events, multiple research has produced varied results about the relationship between financial development and environmental quality. Research has shown that the advancement of financial systems has a crucial role in improving the quality of the environment by reducing environmental degradation.

The article "Exploring the link between economic policy uncertainty, financial development, ecological innovation and environmental degradation; evidence from OECD countries" was retracted in 2025. Reasons: unreliable results or conclusions; concerns about the article.

The governments of OECD countries have implemented their pledges and substantial resources to safeguard the ecosystem and human health from pollution, as well as prevent further environmental degradation [15]. Technological innovation is considered a significant and ideal strategy for achieving both economic growth and environmental protection. Existing literature suggests that the creation and spread of technology advancements not only reduce the increasing pressures on the ecosystem but also maintain an acceptable cost for doing so [16, 17]. Nevertheless, the ecology may suffer negative consequences from technological advancements due to the rebound effect [18]. According to Tanveer et al. [19], the interaction between technical advancements and the diverse characteristics of OECD nations results in a complex and interconnected impact on environmental strategy.

The emissions of only CO_2_ were affected by a multitude of factors, among them, financial development (FD), utilization of renewable energy (REC), technology innovation (TI) and the economic policy (GDPX) of a country. As such, earlier studies have connected FMI, FDI, RECs, TI, as well as GDP [20, 21]. These metrics are essential for long-term, equitable growth in any economy. The expansion of long-term financial resources aids economic expansion. Carbon emissions could rise, which could have either beneficial or harmful effects on the ecosystem [22]. While keeping technological advancement and economic growth under control worldwide, Tanveer et al. [23] investigated the long-term and causative consequences of FD and REC on ecological sustainability. Empirical data from causality testing supported the hypothesis that the variables are related over the long term. Long-term environmental sustainability also benefited greatly from global financial development and the REC. However, Aslam et al. [24] found that economic progress considerably contributes to limiting CO_2_ emissions via efficient energy use.

This study adds to the scientific literature in several important ways: The top environment-polluting OECD countries from 2003–2021 are analyzed to determine the influence of EPU and FD on environmental degradation (ED). However, one of the most pressing concerns we must address is the need for more research into the effects of institutional quality and ecological innovation on the environmental performance of OECD economies. To improve the effectiveness of renewable energy sources, we need the backing of ecological innovation and sound EPU. Considering the OECD countries regarding environmental degradation, it is vital to comprehend the dynamic link between the variables; results add empirical results to the previous literature. (ii) We chose OECD counters for their high fossil fuel usage and environmental degradation rate. In particular, no studies have quantified the effect of EPU and FD on environmental degradation in the OECD economies. To better understand the long-term structural shifts in climate change and environmental degradation, our research focused on the OECD countries to examine the roles played by EPU and FD. In addition, the impact of natural resource rents, foreign direct investment, economic growth and trade on ED in OECD economies (iii). We employ various empirical panel econometric techniques to consider the dependence and heterogeneity across nations that use CO_2_ emissions, such as Sequential estimation of the linear panel data model (SELPDM) and the system-GMM. Multiple tests have been used to check the normality of the data. (iv) Finally, the heterogeneous non-panel technique, proposed by Dumitrescu and Hurlin [25], investigates potential causes and effects among the variables. Results help policymakers to set better solutions to reduce environmental degradation.

The article "Exploring the link between economic policy uncertainty, financial development, ecological innovation and environmental degradation; evidence from OECD countries" was retracted in 2025. Reasons: unreliable results or conclusions; concerns about the article.

Here is how the rest of the research is structured: In Section 2, we present our literature review. In Section 3, we describe the theoretical underpinnings and data collection methods. Methodology frameworks are the focus of Section 4. Section 5 presents the empirical findings and provides commentary on them. A summary and some suggestions for future action are added to Section 6.

## 2. Literature review

CO_2_ emissions cause an environmental threat. The emission of carbon dioxide is an essential factor, among others. The detrimental impacts of CO_2_ on the environment could be mitigated with the help of technological progress and innovation. Here, we review many types of research that have studied the link between CO_2_ emissions and things like GDP, financial growth, renewable energy, and EI. For this objective, our study splits the resources into three distinct categories. The first part of this article covered GDP growth, renewable energy, and carbon dioxide emissions. The connections between renewable energy, inventions, and carbon dioxide emissions were examined, as was the connection between financial growth, REC, and CO_2_ emissions.

### 2.1. EPU and environmental degradation (ED)

Economic policy uncertainty may affect how quickly a region or country implements plans to reduce CO_2_ emissions. As a result, research has been done using both time series and panel methods. Abdul et al. [26] used the traditional ARDL on the UK economy to determine EPU’s role in environmental degradation. He did this by adjusting for factors like economic growth and energy consumption, and he found that EPU had negligible negative and positive effects on the environment in the long and short term, respectively. The use of energy had a comparable but more substantial impact on the deterioration of the natural environment. However, wealth has been shown to have a beneficial effect on the ecosystem. However, Abbasi et al. [27] used the innovative enhanced ARDL technique to uncover the influence of EPU on CO_2_ emissions in France and found that it deteriorated environmental quality over time.

The article "Exploring the link between economic policy uncertainty, financial development, ecological innovation and environmental degradation; evidence from OECD countries" was retracted in 2025. Reasons: unreliable results or conclusions; concerns about the article.

Using China as an example, Liang et al. [28] disentangled the impact of EPU on CO_2_ emissions by factoring in the country’s energy consumption and economic development. However, the study found that increased economic expansion and energy use had long-term adverse environmental effects. However, by running the well-known dynamic ARDL simulations [29], we discovered how income, population, energy intensity, and economic arrangement interact with EPU to determine environmental deterioration in China. The result proved that ecological harm can result from unstable economic policies. These factors devastate the natural world, such as money, population, and energy intensity. The research, however, found that economic structure improves environmental performance.

Yuan et al. [30] used stable panel data for 30 provinces between 2003 and 2017 to examine the effect of EPU on CO_2_ emissions and show that it enhances environmental quality. Environmental rules and energy consumption were found to reduce environmental quality. Recent research by Jóźwik et al. [31] observed the impact of EPU on CO_2_ emissions in Chinese cities and concluded that any surge in EPU had a stimulatory effect.

By adjusting for factors including energy consumption and GDP growth, Shi et al. [32] studied EPU’s impact on CO_2_ emissions in 22 OECD nations. Using PMG-ARDL, the researchers showed that EPU causes long-term increases in CO_2_ emissions. However, the analysis found that short-term energy utilization and economic expansion reduce environmental quality. Song et al. [33] used second-generation unit root and cointegration methodologies to investigate the role of EPU in finding the level of ecological quality across the BRICS countries, and they discovered that EPU improves environmental quality. However, the energy system and related technologies hurt ecosystem health.

Boungou and Mawusi [34] looked at the five most polluted economies and found that EPU worsened ecological quality, even after accounting for variables like REC, economic growth, and ecological innovations. However, all of the influencing factors improved environmental quality. Using a GMM model on data from 137 nations, Zhu et al. [35] found that, from 2001 to 2018, economic policy uncertainty slowed down ecological performance. Hasan et al. [36] examined the impact of EPU on CO_2_ emissions in five eastern countries employing a panel dynamic and distinct regression and came to the same conclusion.

The article "Exploring the link between economic policy uncertainty, financial development, ecological innovation and environmental degradation; evidence from OECD countries" was retracted in 2025. Reasons: unreliable results or conclusions; concerns about the article.

### 2.2. Financial development and environmental degradation

The financial sector lends money to other industries, but the terms and conditions of this lending arrangement change from country to country. Due to the availability of large sums of money from the developed and prosperous financial sector, businesses can expand their operations, resulting in increased pollution. Managers’ confidence in their ability to deal with non-systematic risks is bolstered when large sums of money are available. Financial growth is associated with increased CO_2_ emissions, as shown by the study by Liu et al. [37], which found a positive correlation between economic growth and ED. Direct and indirect links between financial development and ED have been examined by researchers such as Saadaoui et al. [38]. Using the GMM method, Huang et al. [39] deduced that development in the insurance segment has an asymmetric connection with CO_2_ emissions, while Yang et al. [40] stated that financial development positively affects environmental degradation.

Instead, research findings were disseminated to support claims that the FDT improves environmental quality. Green finance, as proposed by Wang et al. [41], is thought to have displaced traditional finance by taxing carbon-oriented schemes and assigning funds toward the establishment of low-carbon technologies. A similar investigation was conducted by Atsu and Adams [42], who determined that FD significantly reduces CO_2_ emissions in G20 countries. In reality, countries worldwide are moving their focus from high-polluting to low-polluting projects and prefer cleaner investment solutions to combat climate change [43].

Though developments in technology and foreign direct investment will undoubtedly have their effects, financial growth also has the potential to have a significant bearing on the sustainable energy market. Costs for renewable energy projects tend to be higher than those for conventional ones. They require substantial initial funding, ongoing innovation supported by R&D expenditures, and patient debt resolution strategies [44]. An undeveloped financial system might inhibit the development of renewable energy enterprises even when demand is high, compared to developed financial systems that aid in expanding the renewable energy industry effectively. According to Tsimisaraka et al. [45], a few research projects have examined this issue. As discovered by Apostolakis et al. [46], liberalization through trade and growth are significant drivers of renewable energy consumption in this context. Similarly, Zhu et al. [47] discovered that the primary factor aggravated by renewable energy consumption in India from 1971 to 2015 was the impact of economic and monetary expansion. These results also imply that a country’s or region’s developed financial position might provide money for transitioning away from renewable energy businesses and toward nonrenewable ones.

The article "Exploring the link between economic policy uncertainty, financial development, ecological innovation and environmental degradation; evidence from OECD countries" was retracted in 2025. Reasons: unreliable results or conclusions; concerns about the article.

### 2.3. Ecological innovation (EI) and environmental degradation

The ability of a country to innovate ecologically is crucial to ensuring a smooth transition from a polluted to a clean environment. To this end, Syed et al. [48] examined technical innovation’s role in determining CO_2_ emissions in Malaysia while also considering GDP growth and the state of the country’s finances. The result validated the negligible impact of technological progress on carbon dioxide emissions. Despite validating the EKC hypothesis, financial progress slows environmental deterioration. Similar results were found in a study conducted by Li et al. [49], who used the traditional Toda Yamamoto and ARDL to investigate the role of EI in determining CO_2_ emissions in Malaysia. They discovered that while income and its square positively affected carbon emissions, EI had a negative effect on environmental quality. Ozcelebi and Izgi [50] implemented innovative strategies for analyzing data panels, such as the AMG and CCEMG estimation strategies. Nuclear and renewable power are excellent for environmental protection. Developing technologies, depleting natural resources, and using nonrenewable energy are all detrimental to the planet.

Nguyen [51] conducted a wavelet effect evaluation of technical innovation and the REC on ED in Portugal and found that technological innovation slows down environmental degradation while using renewable energy speeds it up. FD stimulates ED for both proxies, according to the latest study led in Pakistan by Kim and Yasuda [52], who used novel dynamic ARDL simulations to determine the impact of EI and economic growth on measures of environmental degradation proxied by consumption and territorial emissions. However, this study’s findings show that ecological innovation can slow down environmental degradation.

The relationship between ecological innovation and the environment has been the subject of cross-national research, although no definitive conclusions have been reached. Using the STIRPAT paradigm, Wu et al. [53] studied the connection between ecological innovation and economic growth in BRICS countries. The research, which relied on a static panel design, found that environmental innovation affects ecosystem health. However, the results showed that economic development negatively influences ecological quality. To further investigate the direct and moderating influence of EI on CO_2_ emissions and to untangle the negative heterogeneous effect of EI on CO_2_ emissions, William and Fengrong [54] conducted a panel quantile regression study of 35 OECD countries. The study also showed that using and investing in RE sources is good for the environment.

The article "Exploring the link between economic policy uncertainty, financial development, ecological innovation and environmental degradation; evidence from OECD countries" was retracted in 2025. Reasons: unreliable results or conclusions; concerns about the article.

Using an AMG and a CCMG, Mokni et al. [55] investigated the influence of EI, REC, and institutional quality (IQ) on CO_2_ emissions in 25 African nations. They found that all three factors improve environmental quality. However, wealth, nonrenewable energy usage, and institutional quality confirmed a negative influence on environmental quality. Similar research conducted not too long ago by Han et al. [56] using non-linear ARDL found that the negative shock of EI stimulates CO_2_ emissions in the long run, along with its effects on renewable energy use and export quality. The use of renewable energy sources, however, was proven to boost environmental quality. The findings also demonstrated that adverse shocks slow down CO_2_ emissions while positive shocks speed them up.

### 2.4. Research gap

Previous research disentangled the interplay of the variables and found contradictory results in the field of environmental economics. Notably, only a handful of research studies have examined how EPU and ED affect ED in the OECD economies, and those have yet to find mixed results. Therefore, this research fills a gap in the existing literature by using EPU as a lens to investigate the interconnectedness of the transition to natural resource rents, ecological innovation, institutional quality, trade, economic growth and CO_2_ emissions in the OECD countries. A systematic literature review shows that most OECD economic studies utilized bootstrap ARDL, ARDL, nonlinear ARDL, quantile ARDL, advanced decoupling model, GMM, and bootstrap rolling window causality with various environmental components. This research, however, diverges from past OECD nations’ investigations by using the Sequential estimation of the linear panel data model [57] and the modified version of system-GMM [58]. Since this method can pinpoint instances of cointegration precisely, it was favored. Endogeneity, autocorrelation, and slight sample bias are all manageable. Finally, the study offered policy recommendations geared at SDGs 7 and 13 to fill the gaps.

The article "Exploring the link between economic policy uncertainty, financial development, ecological innovation and environmental degradation; evidence from OECD countries" was retracted in 2025. Reasons: unreliable results or conclusions; concerns about the article.

## 3. Data collection and analysis

### 3.1. Data collection

This study aims to observe the impact of EPU and FD on carbon emissions in 35 OECD economies. The panel data was collected from 2003 to 2021. The control variables are ecological innovation, institutional quality, FDI, trade, and economic growth (See Table 1 & Fig 1).

**Fig 1:** Graphical abstract.

**Table 1:** Description of the variables.

Symbols	Variables	Description	Source
ED	Environmental degradation	Metric tons per capita CO_2_ emission	WDI
EPU	Economic policy uncertainty	World uncertainty index	WUI
FD	Financial development	Bank lending to the domestic private sector as a proportion of GDP	WDI
EI	Ecological innovation	Quantified by the number of trademark applications	WDI
IQ	Institutional Quality	Institutional quality index	WGI (World governance indicator)
GDP	GDP growth	GDP growth (annual %)	WDI
NRR	Total natural resource rent	Total natural resource rents (% of GDP)	WDI
FDI	Foreign direct investment	Net FDI Inflows, as a Percentage of GDP	WDI
TR	Trade	The volume of total trade, % GDP	WDI

Degradation of the natural environment serves as the dependent variable here. Because CO_2_ emissions mirror the primary pollutant emissions and are accountable for roughly 75% of ED [59], CO_2_ is employed as a proxy variable for this phenomenon. In addition, CO2 emissions are a significant contributor to climate change. Due to their polluting nature, these emissions are frequently employed as a proxy for environmental degradation, with EPU viewed as a separate factor. In line with [60], we use the EPU index proposed by Ozkan et al. [61] to create the annual EPU measure by averaging the monthly EPU indexes over a year. We use the natural logarithm of EPU (lnEPU) to maintain uniform dimensions across all metrics. Many existing studies use not only the measure proposed by Arbatli Saxegaard et al. [5] but also the EPU indices proposed by Gregoriou et al. [62]. We also build alternate measures of EPU for robustness tests, modelling our work after [63].

#### 3.1.1. Ethical approval and consent to participate

The authors declare that they have no known competing financial interests or personal relationships that seem to affect the work reported in this article. We declare that we have no human participants, human data or human tissues.

### 3.2. Empirical estimation techniques

CO_2_ emissions are used as a dependent variable in the design of the empirical investigation. Indicators of control variables, including GDP growth, trade, energy consumption, and FDI, are moderated by the independent variables of EPU and the financial development index.

The following equations define the econometric model and the research function:

$$CO_{2}=\int \left(EPU,FD,EI,IQ,FDI,GDP,NNR,TR\right)$$ (1)

In this work, we used a linear version of a static and dynamic panel regression model that links CO_2_ emissions to EPU, FD, ecological innovation, and control indicators:

$$\begin{array}{ll} CO_{2it} & =\alpha_{\text{i}}+\lambda \text{t}+\beta_{1}EPU_{it}+\beta_{2}FD_{it}+\beta_{3}{\text{EI}}_{\text{it}}+\beta_{4}{\text{IQ}}_{\text{it}}\\ & +\beta_{5}FDI_{it}+\beta_{6}GDP_{it}+\beta_{7}NNR_{it}+\beta_{8}TR_{it}+\varepsilon_{it} \end{array}$$ (2)

Where in Eqs 1 and 2, CO_2_, EPU, FD, IQ, EI, GDP, NRR, FDI, and TR represent carbon emissions, economic policy uncertainty, financial development, institutional quality, ecological innovation, economic growth, natural resource rent, foreign direct investment and trade. Further, *αi*, the country-specific effect, from 1–8, shows the coefficients of cross-pending independent variables, and *εit* reports the error term.

The article "Exploring the link between economic policy uncertainty, financial development, ecological innovation and environmental degradation; evidence from OECD countries" was retracted in 2025. Reasons: unreliable results or conclusions; concerns about the article.

By combining Eqs 3 and 4, we get the assessment equation for moderating effects*:

Moderation effects; *EPU* * *EI*, *FD* * *EI on CO*_2_ and *EPU* * *IQ*, *FD* * *IQ* on *CO*_2_

$$CO_{2i,t}=\int \left(\begin{array}{c} EPU,FD,EI,IQ,EPU*EI,FD*EI,\\ FDI,GDP,NRR+TR \end{array}\right)$$ (3)

$$\begin{array}{ll} CO_{2i,t} & =\alpha_{\text{i}}+\lambda_{\text{t}}+\beta_{1}EPU_{it}+\beta_{2}FD_{it}+\beta_{3}EPU_{it}*EI_{it}\\ & +\beta_{4}FD_{it}*EI_{it}+\beta_{5}EPU_{it}*IQ_{it}+\beta_{5}FD_{it}*IQ_{it}+\sum_{j=1}^{k}\;\delta_{j}Z_{jit}+\varepsilon_{\text{it}} \end{array}$$ (4)

Eq 5 displays SELPDM and SYS-GMM estimates.


$$\begin{array}{ll} CO_{2i,t} & =\alpha_{\text{o}}+\alpha_{1}CO_{2_{I,t-1}}+\beta_{1}EPU_{it}+\beta_{2}FD_{it}+\beta_{3}EPU_{it}*EI_{it}\\ & +\beta_{4}FD_{it}*EI_{it}+\beta_{4}EPU_{it}*IQ_{it}+\beta_{5}FD_{it}*IQ_{it}+\sum_{j=1}^{k}\;\delta_{j}Z_{jit}+\varepsilon_{it} \end{array}$$ (5)

#### 3.2.1. Cross-sectional dependency-CD

Conventional methods cannot deal with cross-sectional dependency and heterogeneity, which has a substantial impact on the section on suitable econometric procedures. Therefore, we applied CSDT according to Pesaran et al. [64], Pesaran et al. [65], and Pesaran et al. [66]; the following equations have been carried out for the test statistics.


$$LM=T\;\sum_{i=1}^{N-1}\;\sum_{j=i+1}^{N}\;{\hat{\rho }}_{IJ\underset{d}{\to }X^{2}N\left(N+1\right)2}$$ (6)

$$CD_{lm}=\sqrt{\frac{N}{N\left(N-1\right)}}\sum_{I=1}^{N-1}\;\sum_{J=i+1}^{N}\left(T{\hat{\rho }}_{ij}-1\right)$$ (7)

$$CD_{lm}=\sqrt{\frac{2T}{N\left(N-1\right)}}\sum_{I=1}^{N-1}\;\sum_{J=i+1}^{N}\left({\hat{\rho }}_{ij}\right)$$ (8)

$$CD_{lm}=\sqrt{\frac{2}{N\left(N-1\right)}}\sum_{I=1}^{N-1}\;\sum_{J=i+1}^{N}\left(\frac{\left(T-K\right){\hat{\rho }}_{ij}^{2}-u_{Tij}}{\upsilon_{Tij}^{2}}\right)\left(N,0\right)$$ (9)

The article "Exploring the link between economic policy uncertainty, financial development, ecological innovation and environmental degradation; evidence from OECD countries" was retracted in 2025. Reasons: unreliable results or conclusions; concerns about the article.

#### 3.2.2. Unit root test

Due to their ability to document the variables’ integration order and solve the CSD problem, second-generation panel unit root tests have replaced traditional ones. We used the framework provided by Pesaran et al. [67], commonly referred to as CIPS and CADF, for stationary experiments. To get the test statistic for the null hypothesis test, one uses the following formula:

$$CO_{2i,t}=\alpha_{\text{it}}+\beta_{i}x_{it-1}+\rho_{i}T+\sum_{j=0}^{n}\;\theta_{\text{it}}\;\Delta \;x_{it-j}+\varepsilon_{it}$$ (10)

$$CIPS=N^{-1}\sum_{t-1}^{N}\;\partial_{i}\left(N,T\right)$$ (11)

Where *∂*_*i*_ (*N*, *T*) explains CADF’s test statistics and can be substituted as follows:

$$CIPS=N^{-1}\sum_{i-1}^{N}\;CADF$$ (12)

#### 3.2.3. Westerlund panel cointegration

We analyzed the data to estimate if there is a potential long-term association between ED, FD, EPU, GDP, FDI, NNR, TI and EI. Then, we implemented the target model to explore the effects of independent variables on dependent variables. We use the cutting-edge PCT proposed by Westerlund et al. [68], which incorporates the CSD and SHT and provides practical estimation for long-run cointegration. Long-run cointegration requires the use of the following equation.


$$\begin{array}{ll} \Delta Z_{it} & =\beta_{i}^{\prime }d_{i}+\rho_{i}\left(Z_{i,t-1}-\beta_{i}^{\prime }W_{i,t-1}\right)+\sum_{r=1}^{p}\;\gamma_{i,r}\Delta Z_{i,t-r}\\ & +\sum_{r=0}^{p}\;\zeta_{i,j}\Delta W_{i,t-r}+\epsilon_{i,t} \end{array}$$ (13)

The following equation can be used to derive two sets of statistics from the WECPCT: test statistics for groups (*GT*&*Gα*) and panel statistics (*PT*&*Pα*).


$$G_{T}=\frac{1}{N}\sum_{i-1}^{N}\;\frac{\zeta_{i}}{SE\zeta_{i}}\;;\;G_{a}=\frac{1}{N}\sum_{i-1}^{N}\;\frac{T\zeta_{i}}{\zeta_{i}\left(1\right)}$$ (14)

$$P_{T}=\frac{\zeta_{i}}{SE\zeta_{i}}\;;\;P_{a}=T\zeta_{i}$$ (15)

#### 3.2.4. Dumitrescu and Hurlin causality test

The heterogeneous panel causality test (henceforth D-H) proposed by Dumitrescu and Hurlin [25] is also used to investigate potential causal relationships between variables. Despite the presence of CD, this modified version of the panel Granger causality test yields the same results every time [69]. Here is a rundown of the D-H test’s protocol:

$${\text{W}}_{\text{N},\text{T}}^{\text{HNC}}=\frac{1}{\text{N}}\sum_{\text{i}=1}^{\text{N}}\;{\text{W}}_{\text{i},\text{t}}$$ (16)

$${\text{Z}}_{\text{N},\text{T}}^{\text{HNC}}=\sqrt{\frac{\text{N}}{2\text{K}}}\left({\text{W}}_{\text{N},\text{T}}^{\text{HNC}}-\text{K}\right),\;\text{N}\;\left(0,\;1\right).$$ (17)

where W_i,t_ is the Wald statistic for a given set of data. We can, however, average all Wald static cross sections to obtain ${\text{W}}_{\text{N},\text{T}}^{\text{HNC}}$. Here are the outcomes of the D-H test, including the null and alternative hypotheses: There are many different types of causation. There is a uniform chain of causation.

The article "Exploring the link between economic policy uncertainty, financial development, ecological innovation and environmental degradation; evidence from OECD countries" was retracted in 2025. Reasons: unreliable results or conclusions; concerns about the article.

#### 3.2.5. SELPDM model and the system-GMM

The research uses a modified version of the dynamic SYS-GMM technique [58]. The SYS-GMM method considers endogeneity and is more effective for panel data with longer-time observations. Therefore, dynamic approaches have been applied to empirical research because they yield stable empirical outcomes across a high N and a finite T. Despite its effectiveness, the two-step GMM estimator may suffer from frequent uncorrected standard errors [70]. An innovative method (i.e., SELPDM [57] addresses this problem. In the second step of the SELPDM method, the first-stage residuals involve different explanatory variables, rendering the standard errors inaccurate. To evaluate the reliability of the chosen tools, we run the Arellano-Bond test for autocorrelation and the Hansen J-test for over-identifying restriction. The dependent variable (bank stability) in the dynamic model is represented as follows, with a period lag:

$$\begin{array}{ll} \text{ln}\;{\text{CO}}_{2ijt} & =\alpha_{0}+\beta_{1}\text{ln}\;{\text{EPU}}_{ijt}+\beta_{2}\text{ln}\;{\text{FD}}_{ijt-1}+\beta_{3}{\text{IQ}}_{ijt}+\beta_{4}{\text{EI}}_{jt}+\beta_{5}{\text{GDP}}_{it}\\ & +\beta_{6}{\text{FDI}}_{jt}+\beta_{7}{\text{NRR}}_{jt}+\beta_{8}{\text{TR}}_{jt}+\emptyset_{j}+\lambda_{t}+\mu_{I}+\varepsilon_{it} \end{array}$$ (18)

Using the two-step GMM approach as a baseline, we estimate Eq (16) with dynamic panel data. We then use the SELPDM method to ensure reliability.

## 4. Results discussion

The variables in this study are based on panel data collected from 2003–2021. Reducing variations in the data and so resolving issues linked to seasonal changes can be accomplished using the widely established panel data method for converting low-frequency to high-frequency data [71, 72]; furthermore, it improves the long-run link examination between dependent and independent variables. The first quarter of 2003 through the fourth quarter of 2021 has been collected as a time series of quarterly data. The natural logarithm is performed on every single factor. Explanations for the three exogenous factors considered in this analysis of CO_2_ emission are provided in Table 2.

**Table 2:** Descriptive statistics.

Variables	Mean	Std.dev	Min	Max
CO_2_	2.967	0.763	0.835	3.426
EPU	4.125	0.524	0.025	5.301
FD	12.368	42.257	−11.310	4.528
EI	2432.1	6547.25	−2.983	31267.9
IQ	2.986	20.35	−2.098	46.729
GDP	6.425	16.527	−9.658	8.56
NRR	2095.05	1169.98	−3.652	7965.51
FDI	68.413	52.674	2.049	346.259
TR	102.36	72.54	0.082	510.2

Table 3 displays the correlation matrix, which shows the relationship between variables. It has been found from the results there is a positive correlation among CO_2_, EPU, FD, FDI, GDP, NRR, and TR, while EI and IQ have a negative correlation with CO_2_ emission.

The article "Exploring the link between economic policy uncertainty, financial development, ecological innovation and environmental degradation; evidence from OECD countries" was retracted in 2025. Reasons: unreliable results or conclusions; concerns about the article.

**Table 3:** Correlation matrix.

	**CO**_**2**_	**EPU**	**FD**	**EI**	**IQ**	**GDP**	**NRR**	**FDI**	**TR**
CO_2_	1								
EPU	0.354*	1							
FD	0.207*	0.478**	1						
EI	−0.574**	−0.525**	0.689*	1					
IQ	−0.387	0.629	0.723**	0.336*	1				
GDP	0.468***	−0.625	0.198**	0.408**	0.716***	1			
NRR	0.608*	0.483*	0.249*	0.652**	0.528**	0.143**	1		
FDI	0.726*	0.296	0.509**	0.483*	0.429***	0.634**	0.312*	1	
TR	0.476*	−0.564	0.4693*	0.474*	0.775**	0.714**	0.278*	0.437*	1

Note:

*p<0.05,

**p<0.01,

***p<0.001

Low correlation coefficients suggest no multicollinearity issue exists. A variable’s lack of multicollinearity can be assured if its VIF is less than ten and its tolerance is more than 0.10. Typically, a model is regarded as having no multicollinearity issues if the coefficient values of any given variable are less than 0.85. Table 4 shows that all of our variables meet the requirements for VIF analysis; hence, multicollinearity is not an issue.

**Table 4:** Multicollinearity test.

Variables	VIF	Tolerance
CO_2_	3.346	0.299
EPU	2.109	0.475
FD	1.689	0.593
EI	3.649	0.275
IQ	1.628	0.615
GDP	1.453	0.689
NRR	1.354	0.739
FDI	2.657	0.377
TRD	1.489	0.672

The CD can occur in panel data regression because of cross-country connections in the same socio-economic linkage, environmental considerations, and other unobserved variables.

The following is a chronological account of the empirical strategy used in this investigation. To begin, we test the data for cross-sectional dependence (CD) to see if shocks in one nation propagate to others, as such shocks can lead to erroneous conclusions if they are associated with explanatory variables. The Breusch-Pagan LM test, the Pesaran LM test, and the Pesaran CD test are three of the most popular CD tests in the literature. These three CD tests are used in this study, and their results are presented in Table 5.

**Table 5:** Results of cross-section dependency test.

Indicators	Breusch-Pagan LM		Pesaran Scaled LM		Bias-corrected scaled LM		Pesaran CD	
	Statistic	Prob	Statistic	Prob	Statistic	Prob	Statistic	Prob
CO_2_	2778.634***	0.000	127.597***	0.000	125.604***	0.000	18.958	0.150
EPU	2010.970***	0.000	69.146***	0.000	67.646***	0.000	23.669***	0.000
FD	1033.016***	0.000	120.249***	0.000	118.341***	0.000	38.043***	0.000
EI	790.909***	0.000	91.924***	0.000	89.818***	0.000	10.315***	0.000
IQ	1035.452***	0.000	102.224***	0.000	100.252***	0.000	8.362***	0.000
GDP	4803.934***	0.000	155.643***	0.000	155.455***	0.000	38.066***	0.000
NRR	3013.191***	0.000	150.684***	0.000	148.842***	0.000	4.033***	0.000
FDI	785.661***	0.000	10.131***	0.000	8.239***	0.000	6.145***	0.000
TR	2115.501***	0.000	94.136***	0.000	93.008***	0.000	20.866***	0.000

Note:

*p<0.05,

**p<0.01,

***p<0.001

Because macro-level panel data frequently violates assumptions like low power and size distortions, testing for CD is now a standard when integrating energy consumption and macro-level data before testing for unit roots. Therefore, we adopt the CD test proposed in [67]. Panel A of Table 6 displays these results, which show that the null hypothesis of weak cross-sectional independence was not supported at the 1% level for any of the variables tested. As a result, the CD test shows a cross-sectional relationship between all variables.

The article "Exploring the link between economic policy uncertainty, financial development, ecological innovation and environmental degradation; evidence from OECD countries" was retracted in 2025. Reasons: unreliable results or conclusions; concerns about the article.

**Table 6:** Panel-unit root test.

Tests	CPIS			CADF		
Indicators	Level	1^st^ difference	Order	Level	1^st^ difference	Order
**CO**_**2**_	−0.564*	-	I(0)	−0.622	2.722***	I(1)
**EPU**	−2.613	−3.978***	I(1)	−3.352	4.837**	I(1)
**FD**	−3.712	−2.878***	I(1)	−2.254	2.711***	I(1)
**EI**	−2.980***	-	I(0)	−1.909*	-	I(0)
**IQ**	−2.766***	-	I(0)	−2.264***	-	I(0)
**GDP**	−4.251***	-	I(0)	−1.906*	-	I(0)
**NRR**	−3.331***	-	I(0)	−2.621***	-	I(0)
**FDI**	−2.828**	-	I(0)	−3.169	4.342*	I(1)
**TR**	−1.615*	-	I(0)	−2.791**	-	I(0)

Note:

*p<0.05,

**p<0.01,

***p<0.001

Panel unit root testing, created under the assumption of cross-sectional independence, is used because all variables contain CD. Therefore, we employ the CADF unit root test proposed by [66], which considers CD and can be used to establish the sequence of variables’ integration. All variables are non-stationary at levels but stationary at first differences, as reported by the CADF unit root test in Panel B of Table 2. The CADF unit root test results suggest a long-run equilibrium relationship among the variables because they are all integrated in the same order (I(1)). As a result, we employ panel cointegration testing and continue with the sequential method.

Table 7 displays the outcomes of the panel co-integration test proposed by Westerlund et al. [73]. The findings validate the model’s cointegrating equations. Thus, the independent dimensions produced in this study have long-term connections with environmental quality indices. Our findings demonstrate that the one-group (GT) and one-panel (PT) tests yield statistically significant results. These results suggest that the variables in our model are cointegrated.

The article "Exploring the link between economic policy uncertainty, financial development, ecological innovation and environmental degradation; evidence from OECD countries" was retracted in 2025. Reasons: unreliable results or conclusions; concerns about the article.

**Table 7:** Westerlund panel co-integration test.

Statistics	Gt	Ga	Pt	Pa
**Values**	−3.948**	−19.463	−7.842**	−9.149
**Z-value**	−2.245	−4.349	−0.178	−2.329
**Robust p-value**	0.041	0.724	0.025	0.573

**Note**:

** shows no co-integration at 5% levels.

The long-run coefficients of the independent indicators are measured using two-step-sequential estimations of the linear panel data model (SELPDM) after a long-run correlation among indicators has been confirmed using the panel co-integration test [73].

The results of the SELPDM model are presented in Table 8, and the results of our two-step GMM (for robustness purposes), connected with empirical relations between EPU and FD on CO_2_ emission and with the conditioning impact of EI and IQ, are presented in Table 9. Each need has its own set of data requirements that must be met. The first step is to confirm the lack of first-order and second-order Arellano and Bond autocorrelation (AR1 and AR2). The second finding was that the instrumental factors had no relationship to the error. Our results are credible and objective, as demonstrated by the Roodman et al. [70] over-identification limitation test, the significance of which is assumed to be small.

**Table 8:** The SELPDM- approach for the linear panel-data model.

Independent variables	CO_2_	CO_2_	EI*EPU	EI *FD	IQ*EPU	IQ*FD
			CO_2_	CO_2_	CO_2_	CO_2_
	I	II	III	IV	V	VI
CO_2_	0.924***	0.617**	0.809***	0.758**	0.354***	0.438*
	(9.045)	(2.514)	(6.524)	(2.509)	(3.990)	(1.365)
EPU	7.589***	5.749**	5.248***		4.501**	
	(11.458)	(2.657)	(7.587)		(2.583)	
FD	0.923***	0.357***		0.786***		0.690**
	(5.247)	(5.526)		(3.997)		(2.968)
GDP	0.009*	0.863***	0.087	0.428**	0.268*	0.947***
	(1.719)	(3.968)	(0.528)	(2.987)	(1.237)	(7.583)
NRR	0.689***	0.0749*	0.578***	0.967***	0.526	0.237
	(7.480)	(1.489)	(9.570)	(5.118)	(0.968)	(0.827)
FDI	0.657**	0.247**	0.529***	0.780***	0.472	0.632*
	(2.859)	(2.479)	(3.897)	(7.547)	(0.254)	(1.901)
TR	0.893**	0.489*	0.587*	0.483***	0.639*	0.352
	(2.236)	(1.367)	(1.057)	(3.924)	(1.523)	(0.991)
EI	−0.986***	−0719**	−0.324*	−0.694***		
	(−9.478)	(−2.965)	(−1.058)	(−7.657)		
EI *EPU			−0.978***			
			(−3.879)			
EI *FDV				− 0.557**		
				(−2.698)		
IQ	−0.953***	−0.587**			−0.826***	−0.968***
	(−7.365)	(−2.987)			(−9.213)	(−3.528)
IQ*EPU					−0.964*	
					(−1.952)	
IQ*FDV						− 0.751***
						(−4.807)
Constant	Yes	Yes	Yes	Yes	Yes	Yes
Obs	629	629	623	619	619	619
S. Period	2003–2021	2003–2021	2003–2021	2003–2021	2003–2021	2003–2021
No, of countries	35	35	35	35	35	35
No of IV	29	29	27	25	25	25
No of time	17	17	17	17	17	17
AR-1	0.0362	0.068	0.042	0.021	0.046	0.023
AR-2	0.764	0.826	0.668	0.564	0.382	0.483
Sargan. T, P-values	0.873	0.972	1.000	0.905	1.000	0.912
Hansen, P-Values	0.482	0.896	0.912	0.683	0.917	0.896

Note:

*p<0.05,

**p<0.01,

***p<0.001

The article "Exploring the link between economic policy uncertainty, financial development, ecological innovation and environmental degradation; evidence from OECD countries" was retracted in 2025. Reasons: unreliable results or conclusions; concerns about the article.

**Table 9:** SYS-GMM, robustness test.

Independent variables	CO_2_	CO_2_	EI*EPU	EI *FD	IQ*EPU	IQ*FD
			CO_2_	CO_2_	CO_2_	CO_2_
	I	II	III	IV	V	VI
CO_2_	0.715***	0.428***	0.615**	0.398*	0.296***	0.179**
	(5.154)	(3.992)	(2.529)	(1.996)	(3.981)	(2.053)
EPU	5.364***	4.289**	7.264***		2.098**	
	(9.015)	(2.547)	(2.587)		(2.689)	
FD	0.852***	0.593***		0.402***		0.675***
	(7.251)	(5.842)		(5.214)		(3.997)
GDP	0.021*	0.153**	0.815	0.987*	0.198**	0.746**
	(1.850)	(2.927)	(0.624)	(1.659)	(2.059)	(2.862)
NRR	0.152***	0.346*	0.089*	0.358**	0.489*	0.382
	(5.810)	(1.993)	(1.928)	(2.620)	(1.563)	(0.567)
FDI	0.110**	0.256**	0.209***	0.419***	0.382	0.461*
	(2.520)	(2.826)	(4.109)	(3.990)	(0.179)	(1.990)
TR	0.368***	0.664	0.589**	0.052***	0.537*	0.289
	(4.098)	(0.995)	(2.957)	(5.210)	(1.890)	(0.150)
EI	−0.946***	−0.658***	−0.352**	−0.089***		
	(−3.998)	(−5.010)	(−2.059)	(−3.892)		
EI *EPU			−0.098***			
			(−5.214)			
EI *FD				−0.352**		
				(−2.581)		
IQ	−0.825***	−0.488**			−0.639***	−0.896***
	(−4.639)	(−0.289)			(−9.528)	(−3.998)
IQ*EPU					−0.996**	
					(−2.928)	
IQ*FD						−0.759***
						(−5.648)
Constant	Yes	Yes	Yes	Yes	Yes	Yes
Obs	629	629	625	629	625	625
S. Period	2003–2021		2003–2021	2003–2021	2003–2021	2003–2021
No, of countries	35	35	35	35	35	35
No of IV	27	27	25	23	27	21
No of time	17	17	17	17	17	17
AR-1	0.046	0.183	0.028	0.010	0.569	0.389
AR-2	0.647	0.896	0.589	0.464	0.289	0.543
Sargan. T, P-values	0.908	0.994	0.849	1.000	0.876	0.993
Hansen, P-Values	0.569	0.948	0.602	0.941	0.864	0.910

Note:

*p<0.05,

**p<0.01,

***p<0.001.

t statistics are in parenthesis.

Using the WUI of OECD economies as a stand-in for EPU, the SELPDM results for Eq 5 are presented in Table 8. The correlation between increased economic policy uncertainty and increased carbon intensity raised in the previous section is intriguing. Two primary factors are at play here: Economic growth has been shown to improve energy use and carbon dioxide emissions. Energy consumption has been a significant factor in the OECD’s economic growth for quite some time. The transition toward low-carbon human life will be severely hampered if economic policy is not sufficiently stable and continuous. This situation will lead to a rise in the concentration of carbon emissions in OECD economies. This is a problem all around the developed world [74], not only in developing nations. Second, the consistency of regional economic policy directly impacts how businesses behave in terms of production and energy use. Enterprises in OECD countries with higher levels of economic policy uncertainty and lower levels of economic policy stability are more likely to rely on high-carbon-density fossil energy sources during average production, as shown by an analysis of enterprise survey data in the Chinese tax survey data conducted by Rakpho et al. [75]. In the long run, this will raise the intensity of carbon emissions in the region’s cities and the total carbon emissions produced by businesses there. A growing body of research implies that increased economic policy uncertainty could improve urban low-carbon transformation and enterprise emissions reduction [76]. OECD needs to be cautious about the considerable modification of economic policies and avoid the negative impact caused by changes in economic policies if they want to reach their sustainable development goal on time [77].

The article "Exploring the link between economic policy uncertainty, financial development, ecological innovation and environmental degradation; evidence from OECD countries" was retracted in 2025. Reasons: unreliable results or conclusions; concerns about the article.

At the 1% significance level, the coefficient of financial development was positive, indicating that economic growth has adverse effects on environmental degradation (ED), as measured by CO_2_ emission and EF, respectively. In contrast to the findings of the study by Zhu et al. [78], ours are consistent with the existing literature [79]. These data suggest that expanding the financial sector has unfavorable environmental effects by producing more carbon emissions. It also shows that the scale of financial intermediation affects carbon emissions more than economic development indices but less than efficiency. The positive correlation between the two demonstrates this. The results show that stock market indices significantly affect carbon emissions but are insufficient gauges of the growth of the financial system.

In addition, there is a positive correlation between resource rent (the amount of money made from already-existing natural resources) and pollution output. Increased resource rent increases CO_2_ emissions by increasing the demand for manufactured goods. According to Lee et al. [80], the resource rent has a beneficial effect on industrial activity, which in turn reduces CO_2_ emissions. In conclusion, EPU favors CO_2_ emissions, whereas political stability has a negative impact. This analysis argues that political stability played a significant moderating influence in reducing pollution emissions during the high EPU era.

Institutional strength has been shown to foster environmental progress. Economic institutions that are both effective and efficient promote environmental conservation by decreasing CO_2_ emissions and increasing ecological stability. Syed and Bouri [81] and Al-Thaqeb et al. [82] corroborate the results of our investigation. Simply put, a reduction of 0.1031 per cent in carbon emissions and 0.1593 per cent in ecological footprint over the long term is the direct effect of a one per cent shift in IQ. The short-term effects of the IQ’s efforts to reduce CO_2_ emissions and the EF are also positive. When comparing the positive impact of GG on environmental progress in the long and short terms, the former is more evident due to the greater elasticity of GG in the long run. One possible explanation is that excellent governance improves environmental quality by preventing social and economic instability caused by environmental degradation. According to Lou et al. [83], strong governance has a catalytic role in economic transition by encouraging industrialization, promoting environmental protection, and reducing carbon dioxide (CO_2_) levels. Good governance’s influence on establishing ecological sustainability can be tracked in two ways: directly and indirectly. Since the rule of law has been shown to affect environmental degradation directly, I propose that society exerts pressure on industries to seriously consider their operational decisions by providing direct guidance and strict instruction centered on ecological rules and penalties for noncompliance. In addition, strong institutions safeguard investor interests and property rights, allowing businesses to maximize profits while minimizing their environmental impact [53, 84, 85].

The article "Exploring the link between economic policy uncertainty, financial development, ecological innovation and environmental degradation; evidence from OECD countries" was retracted in 2025. Reasons: unreliable results or conclusions; concerns about the article.

Fourth, based on EI’s long-term (short-term) coefficients, it’s clear that reducing CO_2_ emission into the ecosystem and ecological footprint will improve the current state of the environment, suggesting that a positive relationship exists between EI and ED. A 1.755% (0.159%) reduction in CO_2_ emissions and 1.469% (0.734%) in the ecological footprint are only two examples of how a 1% shift in EI can boost environmental quality. Using new technologies in the manufacturing process helps to promote environmental sustainability. Technological innovation supports environmental conservation by reducing carbon emissions and safeguarding the ecological balance through waste control.

### 4.1. Robustness test

Table 9 shows the combined effect of independent variables on CO_2_ emission in OECD countries. The interactive groups of variables are EI*EPU and EI *FD and IQ*EPU and IQ*FD. The impact of EI *EPU on CO_2_ emission has been observed. Findings demonstrate that the coefficient is negatively significant between EI and CO_2_ emission at a 1% level. On CO_2_ emission, a negative correlation between EI and EPU has been discovered. In OECD nations, where EI has ecologically beneficial effects on CO_2_ emissions, this suggests that the growth of EI in host nations is a crucial component for EPU outcomes to mitigate CO_2_ emissions [86]. The findings highlight EI’s reciprocal influence on carbon dioxide emissions, which is partially offset by the beneficial side effects of this pollutant. Investment in technological innovation leads to lower CO_2_ emissions, as Tran et al. [87] found.

The article "Exploring the link between economic policy uncertainty, financial development, ecological innovation and environmental degradation; evidence from OECD countries" was retracted in 2025. Reasons: unreliable results or conclusions; concerns about the article.

This study included the interaction term FD* EI into the regression Eq (3) to examine the combined effects of FD and technological innovation on the natural world. If the coefficient of EI is positive, it means that a region’s degree of EI is associated with lower levels of CO_2_ emissions. Because of its role in reducing pollution, technological progress has a beneficial and good effect on the environment. Emissions of GHGs, such as smoke dust and SO_2_ emissions, can be lowered thanks to technological advancement, as stated by Okoyeuzu and Kalu [88]. The results of the current study agree with those of previous studies by Hou et al. [89]. Increasing funding and offering low-cost finance help minimize pollution and encourage environmentally friendly activities in line with the technical effect.

To decipher the meaning of the interaction terms above, we must consider how the interdependencies among the variables affect the ecological consequences of CO_2_ emissions. The study’s primary goal is pinpointing the mediating word as the causal link between the two variables. One may investigate the interplay between the two to show how shifts in economic policy uncertainty influence the connection between EI and CO_2_ emissions. The influence of EI in lowering CO_2_ emissions may increase if EPU diminishes and decrease if EPU rises. To see how alterations in FD affect the link between institution quality and CO_2_ emissions, we might also study the interaction between IQ and FD. There may be a positive correlation between FD and the impact of IQ on lowering greenhouse gas emissions, with the inverse being also true.

In addition, the interaction term IQ*EPU in Table 6 has a negative sign, indicating that IQ moderates CO_2_ emission through EPU. The impact of uncertainty can be lessened by boosting IQ. The country’s atmosphere is improved through IQ’s efforts. Our research looks at how well-established institutions can mitigate the impact of EPU on CO_2_ emissions. Institutional solid structures, rules, and regulations can reduce environmental pollution [90]. This suggests that the ecological cost of higher economic development can be reduced through efficient institutions.

Refer to Table 9 to analyze the effects of the IQ*FD interaction on CO_2_ emission. Statistical analysis reveals a significant adverse impact on CO_2_ emissions. Thus, we have included the interaction term IQ*FD in column (6) to inquire into the conditioning function of IQ on the link between FD and environmental deterioration. The five coefficients of this interaction term will likely be a negative sign. Increased FDI and foreign investment in high-tech industries will result from a more institutionally sound environment favorable to FD. The environmental quality as a whole will suffer as a result. The moderating term IQ*FD is incorporated into the model to account for this interaction. Weak institutions are harmful to the environment, whereas strong institutions improve it in OECD countries. Hence, the coefficient on this interaction term is also predicted to be negative. The results of our robustness analysis support our primary finding (see Table 9).

The article "Exploring the link between economic policy uncertainty, financial development, ecological innovation and environmental degradation; evidence from OECD countries" was retracted in 2025. Reasons: unreliable results or conclusions; concerns about the article.

### 4.2. Dumitrescu and Hurlin causality test

Table 10 shows the test statistics, i.e., the W-stat, for evaluating the directionality of the causation between EPU, FD, GDP, EI, TD, FDI, NRR and ED using the causality framework well-known from [25]. And Zbar-Stat for quick evaluations. The research found a two-way causal relationship (EPU = CO_2_ and FD = CO_2_) between economic growth and environmental degradation. This agrees with the findings of studies by Shabir et al. [91] and Tabash et al. [92] on the relationship between economic policy uncertainty and CO_2_ emissions and financial development, respectively. Ecological innovation and environmental degradation and institutional quality and environmental degradation are both explained by the verified unidirectional causality.

**Table 10:** Results of Dumitrescu and Hurlin panel causality test.

Null Hypothesis	W-Stat	Zbar-Stat	P-Value
EPU to CO_2_	4.627***	5.247	0.000
CO_2_ to EPU	2.436	0.267	0.549
FD to CO_2_	5.214***	6.589	0.000
CO_2_ to FD	4.563***	4.265	0.000
FDI to CO_2_	5.324***	4.235	0.000
CO_2_ to FDI	4.638***	3.657	0.000
GTI to CO_2_	4.089***	3.685	0.000
CO_2_ to EI	4.547***	4.687	0.000
CO_2_ to IQ	5.213***	6.018	0.000
IQ to CO_2_	4.680***	3.894	0.000
GDP to CO_2_	3.347**	2.047	0.040
CO_2_ to GDP	2.824	0.289	0.652
NRR to CO_2_	4.859***	4.863	0.000
CO_2_ to NRR	4.632***	4.987	0.000
TR to CO_2_	5.869***	6.487	0.000
CO_2_ to TR	2.479**	0.285	0.048

Note:

*p<0.05,

**p<0.01,

***p<0.001

## 5. Conclusion and policy implications

Traditional economic expansion has relied heavily on fossil fuels, which produce considerable CO_2_ emissions. However, catastrophic harm to the natural ecosystem has been caused by the fast-increasing volume of anthropogenic CO_2_ emissions due to global warming. This not only threatens humanity’s future but also has dire effects on the environment, particularly biodiversity. One of the major difficulties we confront in the twenty-first century is climate change. Humans have invented renewable energy sources to produce clean, sustainable energy that reduces or eliminates CO_2_ emissions. Renewable energy’s continued growth is essential to resolving the climate crisis. The development of effective solutions to climate change will depend critically on our ability to comprehend the interplay between economic policy uncertainties and renewable energies.

The article "Exploring the link between economic policy uncertainty, financial development, ecological innovation and environmental degradation; evidence from OECD countries" was retracted in 2025. Reasons: unreliable results or conclusions; concerns about the article.

Therefore, we provide empirical evidence showing how EPU affects the use of RE sources. Using panel data for 35 OECD nations from 2003 to 2021, we have employed SELPDM and SYS-GMM techniques to get significant results. The parametric estimators reach the opposite conclusion, predicting decreased renewable energy consumption in the face of increased economic policy uncertainty. The image painted by the non-parametric estimator, indicating a non-linear relationship, is different, though. Non-parametric estimations show a negative correlation between 1998 and 2001, a positive correlation between 2003 and 2009, a negative correlation between 2010 and 2013, and no correlation at all outside of these years.

This study focuses on OECD nations and their climate and sustainable development objectives. Without acting to reduce their emissions of greenhouse gases, countries like OECD nations constitute a severe threat to global warming. This is because manufacturing and industrial activities, which are central to its economy, account for a disproportionately high share of the country’s total fossil fuel use, contributing directly to global warming. When it comes to global carbon emissions, OECD nations have made a major contribution. OECD nations are facing a difficult choice between reducing their carbon emissions and trying to keep their national contribution to emissions at or below 2 degrees Celsius, as both are major contributors to global warming. The Paris Agreement of 2005 included China among the countries that committed to limiting global warming. It is fascinating to explore the best potential approaches and policies to help OECD nations rein in their extreme CO_2_ emissions and reach their climate targets as one follows the complexities of OECD nations’ sustainable development in relation to their economic and environmental performance. Therefore, in order to study OECD nations’s sustainable development, we use a variety of scientific methods (SELPDM and SYS-GMM techniques) in conjunction with a range of instruments (including GDP growth, FD, REC, institutional quality and ecological innovation policies). Our emphasis is on the results of the aforementioned scientific methodologies to ensure lucid presentation and understanding of our findings with linked policies. We use SELPDM and SYS-GMM techniques to examine the trend (rise) of carbon emissions in China over two time periods and find that economic growth through economic activities is a statistically significant predictor of this trend over both periods. The good news is that other chosen instruments (FD, EPU, REC, and ecological innovation policies), as revealed by SELPDM and SYS-GMM approaches, tend to reduce and moderate carbon emissions in China. Therefore, if OECD nations adjust their policy to prioritize effective tools, it has a strong chance of reducing its carbon output. The positive consequence of the chosen tools for OECD nations’ sustainable development is confirmed by similar inferential results using bootstrap Granger causality, which corroborate the findings of NARDL and DOLS. Therefore, there is evidence of a causal relationship between technological progress and economic growth in both directions. The OECD economies and ecological innovation are linked in a causal ring that goes both ways. However, the relationship between renewable energy and innovation and environmental quality is causal in only one direction. Finally, other one-way causal connections were looked into, such as the one connecting technological advancement to renewable energy. The interconnected nature of the chosen instruments demonstrates the centrality of technical progress and renewable power sources in reducing carbon emissions.

The article "Exploring the link between economic policy uncertainty, financial development, ecological innovation and environmental degradation; evidence from OECD countries" was retracted in 2025. Reasons: unreliable results or conclusions; concerns about the article.

The results of these methods indicate decisively that EI, REC, and monetary growth are promising avenues for limiting emissions in OECD economies. Officials in OECD economies must investigate the energy transition (away from fossil fuels and toward more sustainable energy sources) immediately. It is recommended that financial growth be promoted through domestic measures aimed at liberalizing the financial sector. This plan will help free up resources for investments like supporting innovative forms of research and development. The availability of cash for technical improvement throughout the energy sectors means this program will have far-reaching effects. The strategy will also help the public and commercial sectors access the financing they need to invest in renewable energy. The renewable energy industry in OECD nations will grow and thrive as a result. To encourage private and public investment in FD, institutional quality, ecological innovation and REC, government officials should draft liberalization and privatization policies. It was also mentioned that policymakers should practice strategies to maintain environmental sustainability by increasing carbon taxes on production and encouraging industries to replace their outdated, high-carbon-emitting technologies with more sustainable alternatives.

The article "Exploring the link between economic policy uncertainty, financial development, ecological innovation and environmental degradation; evidence from OECD countries" was retracted in 2025. Reasons: unreliable results or conclusions; concerns about the article.

### 5.1. Study limitations and further study directions

Finally, this research is relevant to other emerging economies, especially those in Asia and Africa, and has implications for other nations with economic and environmental performance similar to China’s. The study’s limitations stem from the authors’ decision to conduct their research only in China. A panel study of this nature is strongly recommended, particularly for Asian nations. More research is needed, especially using more up-to-date methods and other useful tools.

## Supporting information

S1 Data (XLSX)

## Abbreviations

**ED**: Environmental degradation
**EI**: ecological innovation
**EPU**: Economic policy uncertainty
**FD**: Financial development
**FDI**: foreign direct investment
**IQ**: Institutional Quality
**NRR**: natural resource rent
**OECD**: Organization for Economic Cooperation and Development
**SDG**: Sustainable development goals
**SELPDM**: sequential processes of the linear panel data model
SYS-GMM: System-Generalized method of moments
**TR**: Trade openness
